# Efficacy of Methylprednisolone plus Azithromycin in the Treatment of RMPP and Its Effect on the Changes of T Lymphocyte Subsets

**DOI:** 10.1155/2022/1833195

**Published:** 2022-04-26

**Authors:** Jun Lv, Fei Fan

**Affiliations:** Department of Pediatrics, The Affiliated Changzhou No. 2 People's Hospital of Nanjing Medical University, Changzhou, China

## Abstract

**Objective:**

To explore and analyze the efficacy of methylprednisolone combined with azithromycin in the treatment of refractory *Mycoplasma pneumoniae* pneumonia (RMPP) and its effect on the changes of T lymphocyte subsets.

**Methods:**

A total of 120 children with RMPP admitted to our hospital from September 2016 to September 2020 were randomized at a ratio of 1 : 1 into the control group (conventional treatment) and the observation group (methylprednisolone plus conventional treatment). Outcome measures included clinical efficacy, symptoms mitigation, changes in inflammatory factors, T lymphocyte subsets, and adverse reactions.

**Results:**

Compared with the control group, the total clinical effective rate of the observation group was higher (*P* < 0.05). The disappearance time of cough, wheezing, pulmonary rales, and X-ray lung shadows in the observation group was significantly shorter than that in the control group after treatment (*P* < 0.05). The serum C-reactive protein (CRP), tumor necrosis factor-alpha (TNF-*α*), and interleukin (IL)-8 levels of the observation group after treatment were significantly lower than those of the control group (*P* < 0.05). Compared with the control group, the observation group had a higher CD4+ value, lower CD8+ value, and higher CD4+/CD8+ value after treatment (all *P* < 0.05). There was no significant difference in adverse reactions between the two groups during treatment (*P* > 0.05).

**Conclusion:**

Methylprednisolone plus azithromycin might serve as an alternative in the treatment of RMPP. It facilitates the mitigation of clinical symptoms and signs and regulates the level of inflammatory factors and cellular immune dysfunction, with good effectiveness and a high safety profile.

## 1. Introduction

Mycoplasma pneumonia is a common respiratory disease with a high incidence in clinical practice, and statistics show that the disease accounts for 10%–40% of all community-acquired pneumonia in children [1]. Previously, the disease was believed to resolve spontaneously and was considered self-limiting. However, the increasing high incidence of refractory *Mycoplasma pneumoniae* pneumonia (RMPP) imposes substantial challenges on clinical treatment. The disease progresses rapidly and may lead to the involvement of the lungs. Complications such as respiratory distress syndrome and respiratory failure may occur in severe cases [2]. Methylprednisolone can be used in various acute infections, immune system disorders, or allergic diseases. It has anti-inflammatory and antiallergic effects, inhibits the proliferation of connective tissue, reduces the permeability of capillary walls and cell membranes, alleviates inflammatory reactions, restrains the formation and release of histamine and toxic substances, promotes the decomposition of proteins into sugar, and diminishes the utilization of sugars. As a reliable drug for the treatment of *Mycoplasma pneumoniae* in the current clinical work, azithromycin belongs to the second-generation macrolide antibiotics, but its efficacy in the treatment of RMPP is modest [3]. Research has reported that the modest or even poor treatment effect of RMPP may be associated with the body's immune response and inflammatory response. Therefore, glucocorticoid treatment is suggested in addition to antibiotics, which exerts a strong inhibitory effect on the inflammatory response and regulating the immune function of the body [4]. Accordingly, methylprednisolone combined with azithromycin was used in the present study for the treatment of RMPP to study its efficacy.

## 2. Materials and Methods

The research was approved by the Ethics Committee of the Affiliated Changzhou No. 2 People's Hospital of Nanjing Medical University, No. CZN297927.

### 2.1. Study Population

A total of 120 children with RMPP admitted to our hospital from September 2016 to September 2020 were randomized at a ratio of 1 : 1 into the control group and the observation group. The control group included 35 males and 25 females, aged 3–8 years, with a mean age of (5.68 ± 1.24) years. There were 38 males and 22 females in the observation group, aged 2–7 years, with an average of (5.60 ± 1.17) years. The baseline data in the two groups were comparable.

Diagnostic criteria: patients with a slow or rapid onset, mostly with fever, except in severe cases usually without obvious signs of infectious toxicity; with violent and persistent cough with irritating dry cough as the initial manifestation and with white mucus, similar to whooping cough in severe cases, usually without dyspnea; with significant interstitial changes with patchy or lamellar infiltrative shadows on chest X-ray with or without pleural effusion; with reduced or normal peripheral blood white blood cell count and increased erythrocyte sedimentation rate; and with positive serum *Mycoplasma pneumoniae* antibodies (MP-IgM) and a rise in serum condensation titer of at least 1 : 32.

Inclusion criteria: all patients with diagnosis conforming to the relevant criteria for RMPP in Practical Pediatrics [5], with an ineffective treatment outcome of macrolide antibiotics for 1 consecutive week, with different degrees of increased lung texture and patchy and slightly high-density shadows with blurred boundaries on X-ray, aged less than 14 years, and the family members of the children signed the informed consent form.

Exclusion criteria: patients with congenital heart diseases, bronchopulmonary diseases, and innate immune diseases; with severe liver and kidney dysfunction; with contraindications to glucocorticoids such as tuberculosis at different sites and peptic ulcers; with allergic reactions to the medication used in the present study; those who cannot cooperate with this experiment; and those who lack clinical data.

## 3. Methods

Both groups were given conventional treatment such as oxygen inhalation, phlegm removal, cough relieving, and body temperature control. The control group was given azithromycin (Northeast Pharmaceutical Group Shenyang NO. 1 Pharmaceutical Co., Ltd., approval no.: H20000197) for antiinfection, at a dose of 10 mg/(kg.d) per time, via intravenous drip for 5 days, and the drug was then given through oral administration for 4 days after a 3-day interval. On the basis of the control group,the observation group was additionally given methylprednisolone (Pfizer Inc., approval no.: H20130301)via injection at a dose of 2 mg/(kg.d), administered in 2 intravenous drips, and the treatment continued for 1 week

### 3.1. Efficacy Evaluation Criteria

The clinical efficacy, disappearance time of main symptoms and signs, changes in inflammatory factors, and T lymphocyte subsets before and after treatment were compared between the two groups, and adverse reactions during treatment were recorded. (1) Efficacy evaluation criteria [6]: cured: the symptoms and signs of wheezing, cough, and pulmonary rales disappeared after treatment, and the results of X-ray examination were normal; markedly effective: after treatment, the above symptoms and signs were significantly mitigated, and lung shadow on X-ray examination disappeared; effective: the above symptoms and signs were relieved after treatment, and the lung shadow on X-ray examination was reduced; ineffective: the above symptoms and signs were not improved or even worsened after treatment. Efficacy = (cured cases + markedly effective cases)/total cases *∗* 100%. (2) The main symptoms and signs evaluation items include cough, wheezing, lung rales, X-ray lung shadows, and the disappearance time was recorded. (3) 5 ml of fasting elbow venous blood was collected from children before and after treatment and centrifugated to obtain serum. Enzyme-linked immunosorbent assay (ELISA) was used to determine the levels of C-reactive protein (CRP, Abcam, ab183029), tumor necrosis factor-*α* (TNF-*α*, Abcam, ab 215188), and interleukin-8 (IL-8, Abcam, ab 289967). (4) After blood sample collection, the levels of CD4+ and CD8+ in peripheral blood T lymphocyte subsets were measured by the indirect immunofluorescence method, and the CD4+/CD8+ value was calculated (The monoclonal antibodies were purchased from Huamei Biologicals, Inc., Mc54236, Mc54399). (5) Common adverse reactions include nausea and vomiting, abdominal pain and diarrhea, rash, and local pain.

### 3.2. Statistical Analysis

SPSS 18.0 statistical software was used for data analyses. Enumeration data were expressed as %, and the *χ*^2^ test was used for the comparison. Measurement data were expressed as mean ± standard deviation (*x* ± *s*), and the *t*-test was used for the comparison. Statistical significance was assumed as *P* < 0.05.

## 4. Results

### 4.1. Comparison of Clinical Efficacy

Compared with the control group, the total clinical effective rate of the observation group was higher, and the difference was statistically significant (*P* < 0.05), as given in Table 1.

### 4.2. Comparison of the Disappearance Time of Main Symptoms and Signs

The disappearance time of cough, wheezing, pulmonary rales, and X-ray lung shadows in the observation group was significantly shorter than that in the control group after treatment (*P* < 0.05), as given in Table 2.

### 4.3. Comparison of Inflammatory Factor Levels

Compared with the control group, the serum CRP, TNF-*α*, and IL-8 values of the observation group after treatment were significantly lower (*P* < 0.05), as given in Table 3.

### 4.4. Comparison of T Lymphocyte Subsets Levels

Compared with the control group, the observation group had a higher CD4+ value, lower CD8+ value, and higher CD4+/CD8+ value after treatment, and the differences were all statistically significant (all *P* < 0.05), as given in Table 4.

### 4.5. Adverse Reactions

There was no significant difference in adverse reactions between the two groups during treatment (*P* > 0.05), as given in Table 5.

## 5. Discussion

RMPP, a refractory respiratory disease, features severe conditions and rapid progression, endangering children's lung function and health [7]. Therefore, effective treatment is crucial for disease control. Currently, the second-generation macrolide antibiotic azithromycin is the mainstay for mycoplasma pneumonia, which can effectively control the progression of the disease and inhibit infection [8].

Studies have shown a significant increase in the levels of inflammatory factors in children with *Mycoplasma pneumoniae* pneumonia due to pulmonary infection. TNF-*α* is a broadly bioactive factor that induces neutrophils release and local inflammatory responses, greatly contributing to the generation and development of airway inflammation. The increased expression of TNF-*α* mRNA and protein in lung monocytes-macrophages at the onset of pediatric mycoplasma pneumonia [9] suggests the involvement of TNF-*α* in the pathogenesis of pediatric mycoplasma pneumonia. T lymphocyte subsets are important cells involved in the regulation of the immune system, and their immune imbalance can lead to further exacerbation of the disease, where CD3+ and CD4+ represent that the total T cell population is significantly underexpressed, while CD8+ as a regulatory suppressor is elevated. Mycoplasma can stimulate the body to cause abnormal immune function and secrete a large number of cytokines through the activation of lymphocytes, among which the release of a series of proinflammatory factors such as IL-6 and IL-8 can further aggravate the inflammatory response [10]. IL-6 is an important cytokine in the inflammatory response, and its overexpression can lead to multiorgan and systemic damage. IL-8 causes inflammatory cells to accumulate and release large amounts of active substances through chemotaxis of neutrophils and T lymphocytes. Its overexpression is associated with tissue damage and reflects the degree of infection and regression of pediatric mycoplasma pneumonia.

However, it has been found that macrolide drugs are predisposed to drug resistance in the long-term treatment of mycoplasma pneumonia, and the effect of single drug use is mediocre and even increase in the incidence of macrolide drug-resistant pneumonia [9]. Methylprednisolone can regulate immune and inflammatory responses through lipid-mediated inflammatory factors, and by increasing the sensitivity of the circulatory system to catecholamines, it can improve the body's tolerance to the toxins released by pathogenic bacteria, reduce the damage, maintain the stability of the internal environment, and mitigate the inflammatory responses [10, 11]. In addition, the addition of methylprednisolone on the basis of azithromycin can also significantly enhance the antiinfective effect through the synergistic effect of the two drugs [12].

The results of the present study showed that methylprednisolone combined with azithromycin in the treatment of RMPP leads to a remarkable clinical efficacy and faster mitigation of symptoms, suggesting a promising efficacy of methylprednisolone combined with azithromycin in the treatment of RMPP, which is highly consistent with previous research [13]. Moreover, the addition of methylprednisolone herein resulted in a significantly lower inflammatory factors level in the children. To the best of our knowledge, the abnormal T lymphocyte subsets are associated with immune disorders, and the monitoring of the number of T lymphocyte subsets is of great significance in the diagnosis and prognosis of patients [14, 15]. Here, methylprednisolone combined with azithromycin resulted in better outcomes in terms of inflammatory responses and T lymphocyte subsets versus conventional treatment, confirming that the addition of methylprednisolone benefits the cellular immune dysfunction and immune response of the body, thereby promoting further alleviation of symptoms and signs. Furthermore, the absence of adverse reactions during the treatment with methylprednisolone suggested a high safety profile of methylprednisolone.

Mycoplasma pneumonia can be classified as “asthma” and “lung paralysis,” and its cause is mostly attributed to the fact that children are not yet full of formal qi and are susceptible to external evil, heat, and phlegm, resulting in congestion of phlegm and heat in the lungs. Therefore, treatment should be based on clearing the lung, relieving cough, calming asthma, and resolving phlegm. The medicinal herbs of Wuhu decoction contain ephedra, bitter almonds, gypsum, and licorice. Ephedra is the monarch drug, which can relieve the symptoms of sweating, promote the lung, and relieve asthma; gypsum is the minister drug, which is pungent and cold in nature, can clear heat and remove annoyance, and relieve asthma and cough; bitter almond is the adjuvant drug, which can promote the lung and relieve cough and phlegm, and licorice is the ambassador drug, which can moisten the lung, relieve cough, dispel phlegm, relieve spasm, and harmonize the drugs. The combination of these herbs can promote lung circulation, clear heat, dissolve phlegm, stop coughing, and relieve asthma.

## 6. Conclusion

Methylprednisolone plus azithromycin might serve as an alternative in the treatment of RMPP. It facilitates the mitigation of clinical symptoms and signs and regulates the level of inflammatory factors and cellular immune dysfunction, with good effectiveness and a high safety profile. The limitations of this study are the absence of long-term follow-up and the inadequate collection of medical data of the patients after discharge. The follow-up period will be extended to obtain more reliable clinical data in future studies.

## Figures and Tables

**Table 1:** Comparison of clinical efficacy between the two groups (*n* (%)).

Groups	*n*	Cured	Markedly effective	Effective	Ineffective	Total

Control group	60	32 (53.33)	18 (30.00)	7 (11.67)	3 (5.00)	50 (83.33)
Observation group	60	30 (50.00)	27 (45.00)	3 (5.00)	0	57 (95.00)
*χ* ^2^						4.227
*P*						0.040

**Table 2:** Comparison of the disappearance time of main symptoms and signs between the two groups (d).

Groups	*n*	Cough	Wheezing	Pulmonary rales	X-ray shadow

Control group	60	8.87 ± 0.60	7.64 ± 1.41	12.06 ± 1.03	9.65 ± 1.24
Observation group	60	7.51 ± 0.65	5.43 ± 1.25	9.07 ± 0.83	6.27 ± 1.35
*t*		11.909	9.085	17.509	14.283
*P*		≤0.001	≤0.001	≤0.001	≤0.001

**Table 3:** Comparison of the levels of inflammatory factors before and after treatment in the two groups.

Groups	*n*	CRP (mg/L)		TNF-*α* (ng/ml)		IL-8 (pg/ml)	
		Before treatment	After treatment	Before treatment	After treatment	Before treatment	After treatment

Control group	60	15.78 ± 3.21	12.13 ± 1.89	8.61 ± 1.54	6.08 ± 1.12	18.46 ± 3.25	13.68 ± 2.11
Observation group	60	15.60 ± 2.75	9.87 ± 1.80	8.72 ± 1.65	4.09 ± 0.77	18.51 ± 3.17	10.25 ± 3.97
*t*		0.330	6.707	0.378	11.341	0.085	5.910
*P*		0.371	≤0.001	0.353	≤0.001	0.466	≤0.001

**Table 4:** Comparison of T lymphocyte subsets levels before and after treatment in the two groups.

Groups	*n*	CD4+ (%)		CD8+ (%)		CD4+/CD8+	
		Before treatment	After treatment	Before treatment	After treatment	Before treatment	After treatment

Control group	60	30.24 ± 2.41	32.40 ± 2.23	25.61 ± 2.21	24.85 ± 2.25	1.18 ± 0.42	1.32 ± 0.23
Observation group	60	30.65 ± 2.77	35.79 ± 2.17	25.33 ± 2.25	23.10 ± 2.41	1.19 ± 0.40	1.55 ± 0.26
*t*		0.965	8.439	0.688	4.111	0.134	5.132
*P*		0.194	≤0.001	0.247	≤0.001	0.447	≤0.001

**Table 5:** Adverse reactions during the two groups of medication (*n* (%)).

Groups	*n*	Nausea and vomiting	Abdominal pain diarrhea	Rash	Local pain

Control group	60	2 (3.33)	4 (6.67)	1 (1.67)	1 (1.67)
Observation group	60	1 (1.67)	5 (8.33)	1 (1.67)	2 (3.33)
*χ* ^2^		0.000	0.000	0.000	0.000
*P*		1.000	1.000	1.000	1.000

## Data Availability

The datasets used to support this study are available from the corresponding author upon request.

## References

[1] Zhang Y. (2019). Effect evaluation and clinical analysis of ambroterol oral liquid Jubei mixture in the treatment of children with bronchopneumonia. *Chinese Medicine and Clinical*.

[2] Yin Y., Wu X. (2019). The application value of C-reactive protein, respiratory pathogen antibodies combined with white blood cell count in the diagnosis of early childhood pneumonia. *China Maternal and Child Health*.

[3] Yan C., Sun H., Zhao H. (2019). Epidemiological characteristics of Mycoplasma pneumoniae infection among hospitalized children in Beijing during the past 10 years. *Chinese Journal of Practical Pediatrics*.

[4] Shuang A., Ma S., Chang H. (2019). Efficacy and safety evaluation of compound glycyrrhizin combined with azithromycin in the treatment of children with Mycoplasma pneumoniae pneumonia. *Chinese Journal of Hospital Pharmacy*.

[5] Yu J., Liu H., Liu Yu (2017). Effect of different treatment timings of fiberoptic bronchoalveolar lavage on the therapeutic effect of refractory Mycoplasma pneumoniae pneumonia. *Hainan Medicine*.

[6] Zhang X., Chen Z., Gu W. (2018). Viral and bacterial co-infection in hospitalised children with refractory Mycoplasma pneumoniae pneumonia. *Epidemiology and Infection*.

[7] Mei G. (2017). Observation on the curative effect of antibiotic de-escalation in the treatment of severe pneumonia in children. *China Maternal and Child Health Research*.

[8] Hou H., Zhang S., Liu W. (2020). Efficacy of methylprednisolone combined with azithromycin in the treatment of refractory mycoplasma pneumonia and its influence on inflammatory indexes in children. *Hainan Medicine*.

[9] Wu H., Ding X., Zhao D., Liang Y. W. (2019). Effect of montelukast combined with methylprednisolone for the treatment of mycoplasma pneumonia. *Journal of International Medical Research*.

[10] Hou S. (2017). Effects of budesonide aerosol inhalation combined with methylprednisolone on cytokine expression and immune function of T lymphocyte subsets in children with mycoplasma pneumonia. *Chinese Journal of Practical Medicine*.

[11] He Y. (2017). Efficacy analysis of roxithromycin and azithromycin dry suspension in children with pneumonia caused by mycoplasma infection. *China Maternal and Child Health Research*.

[12] Zhu Z., Wang J. (2017). Effect and safety of gamma globulin combined with glucocorticoid pulse therapy in the treatment of serum CRP in children with refractory mycoplasma pneumonia. *Chinese Journal of Biochemical Medicine*.

[13] Chen H., Qiao Ya (2018). The effect of budesonide combined with terbutaline atomization inhalation on children with mycoplasma pneumonia and its effect on lung function. *Modern Medicine*.

[14] Tan Z., Yang M. (2017). Clinical efficacy of Yanhuning injection in adjuvant treatment of children with refractory Mycoplasma pneumoniae pneumonia and its effects on immune function and cytokines. *Journal of Practical Cardiovascular and Cerebrovascular Diseases*.

[15] Meng G. (2017). Efficacy analysis of glucocorticoids in the treatment of children with refractory Mycoplasma pneumoniae pneumonia. *Chinese Medicine Guide*.

